This article has been retracted.

# Comparative Analysis of Efficacy and Prognosis of Hemodialysis and Peritoneal Dialysis for End-Stage Renal Disease: A Meta-analysis

**DOI:** 10.1155/2022/6007698

**Published:** 2022-03-19

**Authors:** Jingyuan Lu, Danye Shi, Xinhui Zhao, Minhui Xi, Hualin Qi, Qiang He

**Affiliations:** ^1^Soochow University, Soochow 215000, China; ^2^Department of Nephrology, Pudong New Area People's Hospital, Shanghai 201100, China; ^3^Department of Nephrology, Minhang Branch, Zhongshan Hospital, Fudan University (Institute of Fudan-Minhang Academic Health System), Shanghai 201199, China; ^4^Department of Nephrology, Zhejiang Provincial People's Hospital, Hangzhou 310014, China

## Abstract

**Objective:**

This meta-analysis is aimed at systematically assessing the efficacy and prognosis of hemodialysis (HD) and peritoneal dialysis (PD) in the treatment of end-stage renal disease (ESRD).

**Methods:**

China National Knowledge Infrastructure, VIP, SinoMed, Cochrane Library, PubMed, and Embase databases were searched for relevant studies to evaluate the two different dialysis methods for ESRD. The search time was set from 2010 to 2021. Meta-analysis was performed using Stata16.0. The treatment group received PD, while the control group was given HD.

**Results:**

Out of 317 articles initially retrieved, 14 studies were finally included in our meta-analysis. The analysis results showed that there was no marked difference in the 1-year survival rate between the two groups (RR = 1.05; 95% CI: 1.00, 1.10; *P* > 0.05), but the incidence rate of adverse reactions in the treatment group was significantly lower than that in the control group (RR = 0.51; 95% CI: 0.37, 0.70; *P* < 0.05). In addition, PD and HD treatments caused significant decreases in serum creatinine levels (PD, SMD = −2.91; 95% CI: -3.79, -2.04; *P* < 0.05; HD, SMD = −3.09; 95% CI: -4.01, -2.16; *P* < 0.05) and blood urea nitrogen levels (PD, SMD = −2.54, 95% CI: -3.37, -1.72, *P* < 0.05; HD, SMD = −2.62, 95% CI: -3.47, -1.77, *P* < 0.05); however, there was no significant statistical difference in posttreatment levels of serum creatinine and blood urea nitrogen between the two groups. Compared with the control group, the hemoglobin (SMD = 0.56, 95% CI: 0.07, 1.06; *P* < 0.05) and serum albumin (SMD = 1.11, 95% CI: 0.46, 1.76, *P* < 0.05) levels were significantly increased in the treatment group after treatment.

**Conclusion:**

In summary, both PD and HD can improve renal function in uremic patients, but PD is superior to HD in reducing the incidence of adverse reactions, improving the nutritional status, and therefore improving the quality of life of patients.

## 1. Introduction

Uremia, also known as end-stage renal disease (ESRD), is a disease in which chronic renal insufficiency progresses to the terminal stage [1]. This is a metabolic disorder syndrome manifested by an irreversible decline in renal function [2]. Chronic kidney disease (CKD) is the main cause of ESRD. The incidence of CKD in the general population ranges from 10% to 13%, and its prevalence is reported to be 11.5% in some foreign countries [3, 4]. Many patients therefore present with ESRD. ESRD is characterized by long course, high recurrence rate, high mortality, and high morbidity [5]. When CKD occurs in the body, the levels of a variety of substances in protein metabolites, bacterial metabolites, and middle molecular substances are higher than the normal values [6]. At the same time, some substances have toxic effects, resulting in lesions in the digestive system, heart, and lung and causing decreased immunity and high probability of complicating infection [7]. Most uremic patients are in a microinflammatory state, and microinflammatory response has been reported to be closely associated with the progression and complications of ESRD and even the death of uremic patients [8, 9].

Dialysis is an option for ESRD patients who are unable to undergo renal transplantation, which can replace renal function to prolong life [10]. At present, peritoneal dialysis (PD) and hemodialysis (HD) are the two main forms of dialysis treatment [11]. Studies have suggested that PD may be a more physiological form of renal replacement therapy as compared to HD [12]. Some other studies have also reported that in the treatment of ESRD, both PD and HD can stimulate red blood cell phagocytosis, thereby promoting anemia in patients [13]. Different dialysis methods can have different effects on ESRD patients, but there is insufficient evidence regarding these differences. Therefore, this meta-analysis is aimed at systematically evaluating the efficacy and prognosis of HD versus PD in the treatment of ESRD.

## 2. Materials and Methods

### 2.1. Literature Retrieval

China National Knowledge Infrastructure, VIP, SinoMed, Cochrane Library, PubMed, and Embase databases were searched for relevant randomized controlled trials (RCTs) published between 2010 and 2021. The following search syntax was used: (“hemodialysis” and “peritoneal dialysis”) and (“uremia” or “end-stage renal disease” or “ESRD”).

### 2.2. Exclusion Criteria

The exclusion criteria were as follows: (1) review, conference paper, abstract, and case report; (2) uncontrolled before-after study; (3) literature with missing basic data; and (4) duplicated literature, systematic review, and animal experiment.

### 2.3. Inclusion Criteria

The literature included in this meta-analysis had to conform to the following criteria: (1) study subjects: patients with clinical diagnosis of ESRD due to kidney disease; (2) interventions: the control group received HD, while the treatment group was given PD; (3) outcome measures: 1-year survival rate, incidence of adverse reactions, renal function indicators including serum creatinine (sCr) and blood urea nitrogen (BUN) and nutritional status indicators including hemoglobin (Hb) and serum albumin (sALB) before and after treatment, and incidence of dialysis complications (hypoalbuminemia, cardiovascular and cerebrovascular lesions, peritoneal infection, etc.).

### 2.4. Literature Screening and Quality Evaluation

All abstracts and studies extracted from the database retrieval were independently reviewed by two authors. The following data were collected from the selected studies: name of the first author, year of publication, number of patients in each group, study design, and main outcome measures results. The final selection of the studies was jointly decided by two reviewers. In case of different opinions, the disagreement could be resolved through discussion between the two or by a third party's decision. For duplicate reports or extending reports, the ones that had complete data or were published recently were selected. Eligible literature was assessed for quality according to the Newcastle Ottawa Scale (NOS) [14].

### 2.5. Statistical Analysis

According to the Cochrane standards, the data in each included study were combined and then statistically analyzed using Stata 16.0. Heterogeneity of the included studies was assessed using *I*^2^ statistics. *P* > 0.1 and *I*^2^ < 50% indicated no significant heterogeneity among the studies, so a fixed-effect model was used for meta-analysis; otherwise, a random-effect model was adopted for analysis. The results of continuous variables were evaluated using weighted mean difference (SMD), while odds ratio (RR) and 95% confidence interval (CI) weighted the results of categorical variables. Funnel plots were used to assess the publication bias of the studies, and Begg's test was adopted to verify the presence of publication bias when necessary. *P* < 0.05 was considered to indicate a significant difference.

## 3. Results

### 3.1. Literature Retrieval Results

A total of 317 articles were initially retrieved, and then, 262 duplicated articles were removed. Subsequently, 32 articles were excluded by titles or abstracts. After further reading the full-text, we excluded 7 articles with insufficient data and 2 articles irrelevant to uremic patients. Finally, 14 articles were included [15–28].  Figure 1 shows the diagram for the study selection. Data extraction was performed in these 14 included articles, and the baseline characteristics of each included study were shown in Table 1. The NOS scores ranged from 6 to 9, confirming the high methodological quality of the included studies.

### 3.2. Survival and Incidence of Adverse Reactions after Dialysis Treatment

Five articles [15–17, 21, 23] compared patient survival after dialysis treatment between the treatment and control groups. There was no evidence of heterogeneity with *I*^2^ = 0.0% and *P* = 0.742, so a fixed-effect model was used to pool the effect sizes. The results showed no significant difference in the survival rate between the two groups (RR = 1.05; 95% CI: 1.00, 1.10; *P* > 0.05) (Figure 2(a)).

Nine studies [15, 16, 21–25, 27, 28] reported the incidence of adverse effects after treatment. Marked heterogeneity was identified (*I*^2^ = 78.3%, *P* ≤ 0.001), so a random-effect model was used to pool the effect sizes. The results revealed that the incidence of adverse reactions in the treatment group was significantly lower than that in the control group (RR = 0.51; 95% CI: 0.37, 0.70; *P* < 0.05) (Figure 2(b)).

Due to heterogeneity among the included studies, a sensitivity analysis was required. The results showed that the pooled result of the included studies did not change much and the sensitivity was low, suggesting that the results on these two indicators were relatively stable and reliable (Figures 3(a)–3(b)).

### 3.3. Comparison of Blood Urea Nitrogen and Serum Creatinine Levels before and after Dialysis Treatment

Ten articles [17, 18, 20, 22–28] reported changes in BUN before and after PD treatment. The random-effect model was used to pool effect sizes (*I*^2^ = 95.1%, *P* ≤ 0.001) and showed that BUN levels were significantly lower after PD as compared to before treatment (SMD = −2.54; 95% CI: -3.37, -1.72; *P* < 0.05) (Figure 4(a)).

Ten articles [17, 18, 20, 22–28] compared BUN levels before and after HD treatment. There was significant heterogeneity among the studies (*I*^2^ = 95.7%, *P* ≤ 0.001), so a random-effect model was employed for pooling effect sizes and showed that BUN levels were significantly downregulated after HD (SMD = −2.62; 95% CI: -3.47, -1.77; *P* < 0.05) (Figure 4(b)).

Twelve articles [17–28] compared sCr levels before and after PD treatment. By using the random-effect model (*I*^2^ = 96.3%, *P* ≤ 0.001), the results showed that PD markedly decreased sCr levels (SMD = −2.91; 95% CI: -3.79, -2.04; *P* < 0.05) (Figure 4(c)).

Twelve articles [17–28] reported sCr levels before and after HD treatment. The random-effect model (*I*^2^ = 96.9%, *P* ≤ 0.001) revealed that sCr levels were significantly lower after HD treatment compared with those before treatment (SMD = −3.09; 95% CI: -4.01, -2.16; *P* < 0.05) (Figure 4(d)).

The levels of sCr and BUN were further compared between the two groups after treatment. Twelve articles [17–28] compared changes in sCr levels after PD and HD treatments. Due to the evidence of heterogeneity (*I*^2^ = 96.3%, *P* ≤ 0.001), a random-effect model was used to pool effect sizes and showed no significant difference in posttreatment sCr levels between the two groups (SMD = −0.10, 95% CI: -0.40, 0.19; *P* > 0.05) (Figure 5(a)).

Ten studies [17, 18, 20, 22–28] reported changes in BUN after PD and HD treatments. Significant heterogeneity was identified among the included studies (*I*^2^ = 96.9%, *P* ≤ 0.001), and a random-effect model was employed for pooling effect sizes. The results showed that there was no significant difference in posttreatment BUN level between the two groups (SMD = 0.12; 95% CI: -0.26, 0.49; *P* > 0.05) (Figure 5(b)).

Sensitivity analyses were performed due to heterogeneity among the included studies. The analysis results showed that the pooled effect sizes did not change much and had low sensitivity, suggesting that the above results were relatively stable and reliable (Figures 6(a) and 6(b)). In addition, each funnel plot was in a basically symmetrical manner, suggesting small publication bias of the studies included in the two meta-analyses and the reliability of the analysis results (Figures 7(a) and 7(b)).

### 3.4. Comparison of Blood Indexes after Dialysis Treatment

Seven articles [18, 19, 23–27] reported Hb levels in the two groups of patients after treatment. The random-effect model for pooling effect sizes (*I*^2^ = 88.3%, *P* ≤ 0.001) showed that PD led to a significant increase in Hb levels as compared to HD (SMD = 0.56, 95% CI: 0.07, 1.06; *P* < 0.05) (Figure 8(a)).

Nine articles [18, 19, 23–28] compared sALB levels in the two groups of patients after treatment. There was significant heterogeneity in the included studies (*I*^2^ = 93.6%, *P* ≤ 0.001), so a random-effect model was used to pool effect sizes. The results showed that PD led to a significant increase in sALB levels as compared to HD (SMD = 1.11; 95% CI: 0.46, 1.76; *P* < 0.05) (Figure 8(b)).

Due to heterogeneity among the included studies, a sensitivity analysis was required. The results showed that the pooled result of the included studies did not change much and the sensitivity was low, suggesting that the results on these two indicators were relatively stable and reliable (Figures 9(a) and 9(b)).

## 4. Discussion

ESRD is an irreversible decline of renal function when various kidney diseases progress to the terminal stage, and its pathological and physiological mechanisms are complex. There are studies propose “glomerular hyperfiltration hypothesis,” “glomerular hypermetabolism hypothesis,” “trade-off hypothesis,” and “uremic toxin hypothesis” [29, 30]. The incidence of ESRD is increasing worldwide, and since the standardized registration of ESRD, its incidence has shown an increasing trend as a whole in China [31, 32]. This disease results in a serious social and family burden. Renal replacement is an effective and traditional therapy for ESRD, but it should not be the first choice in clinical practice due to the scarcity of organ sources, small range of surgical indications, high cost, and high risk [33]. With the continuous improvement of dialysis technology and equipment, HD and PD have great advantages in the treatment of ESRD. The principles of the two dialysis treatments are different, thus leading to different efficacy and resulting complications [34–36]. Generally, each dialysis method has its place in the treatment of ESRD. Relevant studies have shown that both dialysis methods can improve the quality of life of patients, improve the survival rate, and prolong the survival time; there is no significant difference in the effect of the two on the survival time of patients [37–39]. The equipment for PD is simple, which can be operated at home and is easy to be mastered. PD is more effective in the removal of middle molecular substances and occupies less medical resources. Additionally, PD has better protection of residual renal function and has little effect on the body's hemodynamics. By contrast, HD can quickly and effectively remove small molecular solutes and water. Fistula puncture is required for each dialysis, affecting internal environment and hemodynamics of the body and resulting in a faster loss of residual renal function and more contacts to viral infection and medical staff [40, 41].

Systematic searches from the database were performed at home and abroad to identify relevant studies to objectively evaluate the effectiveness of PD and HD in the treatment of ESRD. Finally, 14 controlled studies that met the criteria were selected. There was little difference among these included studies in terms of study subjects, study design, and outcome measures, and these studies had clear inclusion and exclusion criteria and similar baseline characteristics. Therefore, a meta-analysis based on these studies could be carried out.

In this meta-analysis, we found no significant difference in 1-year survival between uremic patients treated with PD and HD. However, the incidence of adverse reactions after PD treatment was significantly lower than that after HD treatment. Jin et al. [16] similarly confirmed that HD patients had a significantly higher incidence of dialysis-related complications in the first 30 days than PD patients and a higher incidence of bacteremia. An increase of sCr and BUN is one of the indicators for the diagnosis of renal injury [42]. In this study, we found that sCr and BUN were significantly lower after treatment regardless of PD or HD. But no significant difference was identified in posttreatment levels of sCr and BUN between the two dialysis modalities. Further, the changes of blood indexes (Hb and sALB) in uremic patients after PD or HD treatment were analyzed; the results showed that PD decreased the occurrence of hypoalbuminemia and anemia compared with HD but improved the nutritional status of patients. This is consistent with the findings of Obrador et al. [43]. They found that patients receiving PD had a lower prevalence and severity of renal anemia than HD patients. Collectively, these above results confirmed that both dialysis methods are effective in treating ESRD, but PD was significantly superior to HD in improving the nutritional status of patients and in decreasing the incidence of clinical adverse reactions.

This study still has the following limitations. First, the quality of studies included in our meta-analysis is limited, and most of them are Chinese studies. Also, the number of included articles is limited. There are few studies regarding long-term efficacy of dialysis treatment, and the sample size included is small. Whether the increase in sample size will lead to changes in the outcome measures still needs further study.

## 5. Conclusion

Both PD and HD can improve renal function and strengthen small molecule removal. However, compared with HD, the levels of Hb and sALB after PD increased significantly, indicating an improvement of the nutritional status of patients. PD is also superior to HD in decreasing the incidence of adverse reactions and therefore improving the quality of life of patients.

## Figures and Tables

**Figure 1:** Literature screening process.

**Figure 2:** Comparison of survival rate and incidence rate of adverse reactions after dialysis treatment between the two groups of ESRD patients. (a) Forest plot of survival rate and (b) forest plot of incidence rate of adverse reactions. ESRD: end-stage renal disease.

**Figure 3:** Sensitivity analysis of survival rate and incidence rate of adverse reactions after dialysis treatment in two groups of uremic patients. (a) Sensitivity analysis of survival rate and (b) sensitivity analysis of incidence rate of adverse reactions.

**Figure 4:** Comparison of blood urea nitrogen and serum creatinine levels before and after dialysis treatment in two groups of uremic patients. (a and b) Forest plots of blood urea nitrogen (BUN) levels before and after peritoneal dialysis (a) and hemodialysis (b). (c and d) Forest plots of serum creatinine (sCr) levels before and after peritoneal dialysis (c) and hemodialysis (d).

**Figure 5:** Comparison of serum creatinine (sCr) and blood urea nitrogen (BUN) levels after dialysis treatment in two groups of uremic patients. (a) Forest plot of sCr levels and (b) forest plot of BUN levels.

**Figure 6:** Sensitivity analysis of serum creatinine (sCr) and blood urea nitrogen (BUN) levels after dialysis treatment in two groups of uremic patients. (a) Sensitivity analysis of sCr levels and (b) sensitivity analysis of BUN levels.

**Figure 7:** Funnel plots of serum creatinine (a) and blood urea nitrogen (b) levels after dialysis treatment in two groups of uremic patients.

**Figure 8:** Comparison of blood indexes after dialysis in two groups of uremic patients. (a) Forest plot of hemoglobin (Hb) levels and (b) forest plot of serum albumin (sALB) levels.

**Figure 9:** Sensitivity analysis of blood indexes after dialysis in two groups of uremic patients. (a) Sensitivity analysis of hemoglobin (Hb) levels and (b) sensitivity analysis of serum albumin (sALB) levels.

**Table 1:** Basic characteristics of the included literature.

Study	Year	Sample time	Cases treat/con	Age (years)		Sex ratio (M/FM)		Study design	Treatment time (months)	NOS	Outcome measures
				Treat	Con	Treat	Con				
Qiu jing	2015	2011.01~2013.02	50/50	51.3 ± 7.8	50.2 ± 8.9	26/24	28/22	RCT	3	6	③④⑤⑥
Qiu junfei	2019	2015.03~2017.03	30/30	46.5 ± 6.6	46.1 ± 6.5	18/12	17/13	RCT	6	7	③⑥
Cui dongfeng	2016	2013~2014	40/40	63.2 ± 13.1	62.4 ± 12.5	23/17	22/18	RCT	6	6	①②③⑤
Tian yuan	2019	2017.01~2018.12	48/48	51.3 ± 8.3	51.3 ± 8.3	29/19	29/19	RCT	3	7	②③④
Zhou pengyu	2021	2018.01~2020.01	40/40	67.1 ± 7.4	66.8 ± 7.5	22/18	24/16	RCT	6	7	②③④⑤⑥
Fu tianwen	2019	2013.04~2018.04	34/34	56.4 ± 14.7	51.5 ± 18.5	17/17	18/16	RCT	6	7	③④
Wang jie	2015	2013.06~2014.08	30/30	42~69	42~69	18/12	18/12	RCT	3	6	③④⑤⑥
Liu jia	2019	2017.01~2017.12	25/25	56.8 ± 3.4	57.2 ± 4.3	13/12	15/10	RCT	6	7	②③④⑤⑥
He laiming	2020	2015.01~2018.12	30/30	61.1 ± 5.7	60.3 ± 5.3	17/13	16/14	RCT	6	7	②③④⑥
Haijiao Jin	2016	2013.01~2014.12	98/82	55.2 ± 17.9	51.2 ± 20	56/40	44/38	RCT	3	8	①②④⑤⑥
Shen yan	2016	2010.01~2013.01	46/48	56.8 ± 14.2	57.8 ± 14.9	29/17	31/17	RCT	6	8	①②③④⑤⑥
Xing an	2014	2012.02~2013.06	52/88	53.1 ± 11.5	52.8 ± 10.2	27/25	51/37	RCT	12	6	②③④⑤⑥
Huang zanwei	2012	2011.05~2012.05	40/40	36~73	37~75	22/18	24/16	RCT	6	6	①③④⑥
Xiujuan Zang	2020	2005.01~2015.12	309/233	73.1 ± 5.6	72.6 ± 7.5	179/130	123/110	RCT	12	8	①②⑥

Note: Treat: Treatment group; Con: control group; M: male; FM: female; RCT: randomized controlled trial; ①: 1-year survival rate; ②: adverse effects rate; ③: serum creatinine; ④: blood urea nitrogen; ⑤: hemoglobin; ⑥: albumin.

## Data Availability

The data used to support the findings of this study are available from the corresponding author upon request.
